# Analytical Study of Financial Accounting and Management Trends Based on the Internet Era

**DOI:** 10.1155/2022/5922614

**Published:** 2022-08-22

**Authors:** Qin Li

**Affiliations:** College of Accountancy, Shanxi Technology and Business College, Taiyuan 030000, Shanxi, China

## Abstract

With the development of Internet technology and computer technology, the network has provided convenience to enterprises while putting forward new requirements for the development of the accounting industry. The combination of traditional financial accounting methods and computerized information technology enables accurate and rapid transmission of financial data. At the same time, the application of network technology optimizes the financial accounting process of enterprises and greatly improves the efficiency of accounting work and accountants can devote more time and energy to the analysis of enterprise financial information. However, with the application of Internet technology, the change in financial accounting has also generated new problems. The article focuses on the topic of financial accounting; first, it briefly introduces the development history of financial accounting and the Internet; second, it discusses the changes in accounting work mode and its characteristics under the network environment and analyzes the advantages and problems of combining network technology and financial accounting; and finally, it puts forward the countermeasures to solve the “Internet+” era financial accounting work for the current situation. Finally, the countermeasures to solve the financial accounting work in the era of “Internet+” are proposed to improve the professional ability of financial personnel.

## 1. Introduction

Compared with the previous enterprise financial management work, financial management in the Internet era has distinct advantages, which effectively expands the scope of enterprise financial management and allows comprehensive supervision of the entire financial management work [1]. In the Internet era, corporate financial management generates more information and requires rapid transmission of information in a short period of time [2]. If they want to meet the development needs of the times, enterprises need to have a clear understanding and awareness of the importance of financial and accounting management work to innovate the working model (Figure 1). At the same time, enterprises also need to improve the dissemination of financial information and manage financial accounting information in a diversified way, which can not only effectively improve the efficiency of enterprise financial management, but also optimize the working environment comprehensively [3]. In the Internet era, intelligence has become the main direction of enterprise financial management work, which is an important basis for enterprise financial management in the Internet era and an inevitable trend of the market economy, which can not only effectively improve the market competitiveness of enterprises, but also facilitate the implementation of scientific management by relevant financial and accounting departments and lay a solid foundation for the efficient development of financial accounting [4]. Therefore, in the Internet era, enterprises need to pay more attention to the informationization and intelligence of financial accounting management, fully meet the development trend of the times, and actively promote the development of enterprises [5].

Nowadays, China has entered the Internet era, and the vigorous development of the Internet has directly changed the financial accounting management work, significantly improved the management quality of financial accounting, and the content involved in financial accounting has become more extensive [6]. For this reason, relevant personnel must deeply analyze the financial accounting management trends in the Internet era in order to do their jobs well.

### 1.1. Expanded Scope of Financial Management

In the Internet era, the management efficiency of enterprises has been significantly improved, and the financial accounting management mode has been changed [7]. The most significant change is that it extends the scope of financial management and enriches the work of financial management. For example, the use of the Internet not only enables direct procurement and management but also the ability to discipline suppliers and later sales to ensure the integrity of management [8].

### 1.2. Improving the Timeliness of Financial Management

Real-time and timeliness are the most significant advantages of Internet technology, so for financial accounting management work, it is also necessary to improve the speed of information transmission to help users get accurate information [9]. Financial and accounting management pays more attention to the timeliness of information, and the existence of Internet technology helps meet this need effectively [10]. The use of Internet technology enables financial management to be more timely and changes the method of communication, increasing communication and exchange between personnel [11]. For example, the use of the Internet makes it possible to lay out the relevant work content and to monitor the implementation of the work; the use of the Internet also makes it possible to give feedback to the company on specific work situations, significantly improving efficiency [12].

### 1.3. Orderly Operation within the Enterprise

Financial accounting management work in the Internet era can deliver financial information in a timely manner and make financial management work more flexible and orderly [13]. Financial accounting management work is the focus of enterprise management. In enterprise financial accounting management, it is difficult to achieve obvious management effects if we still rely on the older way to implement management. At this time, the use of Internet technology can manage the financial and business work scientifically and ensure the orderliness of the internal operation of the enterprise.

At present, China is in the era of intensified economic globalization and extremely rapid transmission of information, and the competition among enterprises is increasingly fierce. In the face of the increasingly competitive market environment, leaders need to conduct enterprise management not only to consider the traditional factors of competition between enterprises, but also to start from the management level, relying on strong and excellent financial management to help managers to make appropriate corporate decisions [14]. Therefore, real-time and comprehensive financial management information plays a pivotal role for managers to make decisions.

## 2. Related Work

Financial accounting is a branch of business accounting that, together with management accounting, forms the two main areas of business accounting, known as “traditional accounting” because it follows traditional manual accounting records, and therefore also known as “external reporting accounting” because it focuses on the business external stakeholders' decision-making needs and financial reporting outside the enterprise [15]. Financial accounting is an economic management activity that is carried out through comprehensive and systematic accounting and monitoring of the financial flows carried out by the enterprise, with the main purpose of providing economic information about the financial position and profitability of the enterprise to external investors, creditors and relevant government agencies that have an economic interest in the enterprise (refer to Figure 2).

Financial accounting plays a pivotal role in enterprise management and can provide useful information to decision-makers through various accounting procedures, actively participate in the management decisions of the enterprise, improve the efficiency of production and operation activities of the enterprise, and promote the healthy and normal development of the market economy. Therefore, financial accounting is crucial and indispensable in the course of the development of enterprises [16].

The Internet was born in the 1960s and 1970s as a large global network consisting of a series of common protocols [17]. As the economy grew, the development of the Internet accelerated, and by the 1980s and 1990s, it had matured, become more sophisticated, and gradually began to spread around the world [18]. Throughout the early development of the Internet, fundamental changes occurred almost every decade [19]. In China, the adoption of the Internet began around 1994 [20].

With the increasing popularity of mobile Internet, cloud computing, big data, and other technologies, human beings have stepped into the Internet era. Whether it is attendance records and online shopping, daily commuting to and from work, or software used in daily work, Internet technology is necessary [21]. It can be seen that technology has a decisive influence on the development of society, and the development of network technology will continue to push human society into a new era.

By applying Internet technology to financial accounting and management, the transport linkage of computer data and automatic calculation of data are realized, which in turn improves the accuracy of financial data in a comprehensive manner [22]. In addition, with the support of Internet technology, workers effectively enhance the degree of information sharing in daily financial accounting or management and create good conditions for the smooth implementation of financial supervision [23]. For example, in daily work, when workers need relevant financial information, they can quickly obtain the required information with the help of information sharing. Although Internet technology has improved the efficiency and quality of financial accounting and management work, the content of financial accounting and management work in the new era is gradually diversified and complicated [24].

With the gradual diversification of financial management content, the financial management staff of institutions can fully understand the importance of this work and continuously improve their Internet technology and financial management knowledge and skills to better meet the needs of the real work, and then give full play to the maximum value of financial management work [25].

## 3. Methodology

### 3.1. Basic Model

An accounting information system (AIS) is a system that incorporates all accounting information. AIS is an important application of computer technology in the field of accounting; the generation of AIS brings accounting from the original era of manual bookkeeping to the era of machine bookkeeping, realizing computerization of accounting is an important reform in accounting practice. Its essence is the use of computers for an accounting information system.

The mechanism of its role is that the accounting information system first collects some of the data produced by the front-end business process that meet the definition of accounting, then carries out corresponding accounting processing according to these accounting data, completes accounting, generates accounting information, and finally, managers use this accounting information to make business decisions. Analysis and organization of the role mechanism of AIS is shown in Figure 3.

In this article, “whether the accounting information system can realize the sharing of business and financial data” is taken as the mark of the division between traditional and financial integration accounting information systems; from this perspective, the traditional accounting information system has gone through five rounds of evolution, as shown in Figure 4.

Although the accounting information system in the first 4 stages could also record some business information, the content of the recording was very limited, and business information still needed to be transferred between business and finance departments through paper-based original vouchers. Compared with the first 4 stages, the most significant feature of this stage is that the front-end business module is incorporated into the AIS, which helps the AIS record not only the business data conforming to the accounting definition, but also other types of business data so that the AIS system provides managers with richer data and enables managers to see the original business picture more intuitively through the system.

Through the above 5 stages of development of an accounting information system, we can see that the traditional accounting information system mainly solves 2 problems: first, for the paperless bookkeeping vouchers, accounting personnel use computers instead of manual bookkeeping; second, recognizing that business data play a very important role in enterprise management, business department data and financial data are integrated into the accounting information system, so that the accounting information system can further play its efficient management role.

Through the above development history of traditional accounting information system, it can be seen that traditional AIS provides accounting information to managers and then provides services for their management decisions, although the MIS (management information system) stage can already provide business information to managers, but because business and financial information cannot be shared resulting in a lower degree of this information used by managers, so by organizing the traditional AIS functions as shown in Figure 5.

Industry financial integration AIS means an accounting information system that can realize business financial integration, which is an effective platform and tool for enterprises to realize business financial integration by using various modern computer technologies, advancing the financial work of enterprises to the business end, through which enterprises can not only obtain management information in terms of financial analysis, but also obtain management-related information directly from business data, and managers can use this business-side information for more in-depth analysis, realizing the integration of information flow and data flow.

The accounting information system of the combination of production and finance realizes the information sharing of business and financial data, breaks through the limitation that traditional accounting information systems basically can only use accounting information to participate in management, improves the utilization of business information, and promotes a deeper combination of accounting and management; the combination of accounting and management makes accounting a powerful assistant of enterprise management. The functions of financial accounting and management accounting are therefore mutually reinforcing and inseparable, as shown in Figure 6.

### 3.2. Improvement Model

Based on the aforementioned problems of rigid accounting, rigid management, and rigid business processes in the application process, the design goal of the flexible financial integration AIS is to make the financial integration AIS flexible, improve the self-adaptability and scalability of the system itself to changes in external requirements, and then shorten the system redevelopment cycle and reduce the cost of redevelopment, specifically including flexible input and data structure, flexible data flow, flexible business process, and flexible data output.

#### 3.2.1. Flexible Input and Data Structure Design

Traditional industry and finance integration AIS for the development of data structure design is usually only specific database tables and fields, that is, the premise that the default later database table structure does not change, the data table in the data items does not change. This rigid system does not take into account the possible adjustment of the data structure in the subsequent use of the enterprise during the initial design, and of course, there is no input space reserved for the user to configure the data structure at the front end, so the developed system lacks self-adaptability for the user to a certain extent in terms of input and data structure.

Two important concepts in the database related to the input and data structure design of the flexible industry financial integration AIS are triggers and stored procedures. The trigger mechanism ensures that the trigger action is executed only when the trigger event occurs and the trigger limits are met. Each table in the database can set a trigger, and the role is to establish the connection of multiple tables in the database to achieve the linkage of data in multiple tables. A stored procedure is a set of statements to complete a specific function, through the parameters set so that when the user performs similar operations on the database, there is no need to repeat the compilation, so the use of stored procedures can improve the efficiency of the database operation.

The design of the data structure in the flexible financial integration AIS is not only the specific database tables and fields, but also the “data dictionary,” which stores not the general specific user data, but the structural data of various data items, and establishes the connection between the data dictionary and the entity database tables through triggers and stored procedures, so that when the structural data in the data dictionary changes, the corresponding entity table structure will also change accordingly.

The design of input in the flexible business financial integration AIS is to present the data dictionary stored in the database on the page to the user by setting up the data dictionary function card interface, reserving the input space for the user to configure the data structure. Using this function, the following two kinds of operations can be performed: first, you can create new original documents and enter the specific data items related to the content; second, you can modify the original documents in the data items (such as special enterprises in financial accounting or managerial decision-making needs may add some special data items on business documents, which you can add or modify in the original database forms) and thus meet the changing needs of enterprises for the data structure.

The “data dictionary” is a “warehouse” that can be used to store a variety of structural data. It should include the following two tables: one is the detail table (to store the content of the data items of each table of the database, including field names and field types), and the table structure as shown in Table 1.

The flexible implementation process of input and data structure is shown in Figure 7. The data update linkage between the business and finance fusion AIS and the corresponding entity tables in the database is done through triggers and stored procedures. When the user performs the operation of adding, deleting, or changing in the data dictionary function card of the AIS, the corresponding database is called using the database interface; the corresponding data changes are recorded in the detail table; the operation of adding, deleting, or changing then triggers the trigger embedded in the detail table; the data modified by the user in the front-end page is recorded in the temporary table; the corresponding stored procedure is executed; and then, the corresponding entity table is modified. The modification of the entity table will be presented on the interface of the AIS in real-time, so that the user can realize the change in the data structure of the corresponding form in the database through the data dictionary function card on the AIS, which realizes the flexibility of the input and data structure.

#### 3.2.2. Flexible Data Flow Design

Since the data structure in the traditional AIS is fixed, the flow of data items between them is also fixed. Although the flow of data items between documents, between documents and vouchers, and between documents/vouchers and reports is possible in the traditional rigid AIS, this flow is solidified and does not allow users to configure themselves, for example, some data grievances exist only in upstream documents and not in downstream documents, but managers need to add these data items that exist only in upstream documents to downstream for management purposes The administrator also needs to add these data items that exist only in the upstream documents to the downstream documents for management purposes. If the new data items do not exist in the upstream and downstream documents, it is difficult to configure the process of these extended data items in the system.

The design of the data flow in the flexible financial integration AIS focuses on the establishment of visualized document conversion rules between upstream and downstream documents, between various documents and vouchers, and between documents and reports, which can be configured by users. The specific design diagram is shown in Figure 8.

Document conversion rules: Document conversion rules are designed to make the data conversion between documents more convenient, and through the method of parameter configuration, the conversion rules are no longer rigid and unchangeable but can be flexibly deployed. With the rules to achieve data filtering, grouping, and merging, calculation and other configurations meet the business needs of the document conversion process. Document conversion rules are broadly divided into single-head conversion rules, entry conversion rules, auxiliary configuration, etc. The parameter configuration through the single-header conversion rules can establish the association of each data item between documents, and the parameter setting in the journal entry conversion rules can realize the reconfiguration of generated vouchers.

#### 3.2.3. Flexible Business Process Design

In the traditional rigid business finance system, due to the fixed setting of business processes, business users cannot adjust business processes according to their actual needs, and the integration of business and financial processes can only set up financial indicators according to business needs, and cannot optimize business processes according to the financial indicators of enterprises, and the setting of business processes can only realize the one-way business process of A-B-C one-way business process. With the large number of business needs of enterprises, the traditional rigid business process structure can no longer meet the needs of the complexity of enterprises today.

The core of business process design in flexible AIS is that users themselves can realize business process customization. Business process customization means that the system provides a common business process model in advance to support users to personalize the operation according to their needs, allowing users to realize the dynamic combination of processes or dynamic definitions without changing the source code, increasing the flexibility of business processes in the financial system. The flexible AIS provides users with the function of freely configuring business processes, and realizes the close connection between business process management and the AIS of financial integration.

The flexibility of business process customization is reflected in the following aspects, and the overall process of its operation is shown in Figure 9.

#### 3.2.4. Flexible Data Output Design

The traditional financial integration system is relatively fixed in the final output report format and content, for example, the format of the four commonly used financial statement templates are relatively fixed, and the content is relatively fixed, so if the project name or data source inside the template report changes, the enterprise cannot change and adjust in time by itself, so the rigid financial integration AIS has caused the limitation of management analysis to a certain extent.

The design of flexible data output in the flexible industry financial integration AIS focuses on the user's ability to configure the content and format of information output, as mentioned above, for the final financial accounting reports and management accounting reports, the manager can choose the output content and format at will, and if the items in the reports defined in the system template do not meet the actual needs, the user can customize the report format and content to meet the personalized needs of managers. Flexible AIS supports customizable report function, which allows users to design the report format, report items, sources, calculation, and processing methods by using the visualized pages provided and combining them with the actual situation of the unit and the department. The system will automatically generate the reports that the user wants according to his or her definition. Once the user's needs change, the user can modify the original report design or design a new report to meet his or her needs without modifying the accounting information system itself. That is, the core of the design of data output flexibility lies in the implementation of the custom report function, the specific design process of which is shown in Figure 10.

## 4. Case Study

A company is a large integrated modern enterprise group. With the gradual expansion of the group's scale, it became difficult to adapt the original financial and business model to the group's management needs, which to a certain extent hindered the group's development. To keep pace with the times, in the context of the Internet, it is imperative to make full use of new information technology tools for reform. We first show the degree of approval of different employees for the management upgrading of the financial accounting system in Figure 11.

Before the implementation of financial sharing, the finance department of a company was mainly responsible for daily accounting, expense reimbursement, current account management, fundraising and operation, investment management, budget management, tax reporting, statement preparation and analysis, and other work, mainly centralized financial management. With the development of a company, the number of subsidiaries, overseas branches, and strategic business units gradually increased, the group reformed and adopted the organizational form of group customer divisions, and established financial divisions within each division; from a centralized financial management mode to a decentralized financial management mode, each divisional financial division is responsible for its own local business corresponding to the expense reimbursement accounting and other work. Then, each business unit regularly sends business-related data to the accounting staff of the business unit, and the accounting department of each business unit submits the processed financial and business analysis data to the headquarters group for data aggregation and analysis.

### 4.1. Analysis of the Main Problems of a Company before the Integration of Industry and Finance

1. *High Labor Cost and Low Value Creation*. A company's customer business units establish the same function as the finance department: repeatedly building a finance department is time-consuming and labor-intensive, and a large number of accounting staff increase the group's operating costs. The heavy accounting volume of each finance department takes up a lot of energy of accounting staff, making it difficult for them to withdraw business management and provide decision support for business strategy management.
2. *Poor Information Communication*. First of all, a company arranges accounting personnel with the same functions in different group customer divisions, and the financial information is first aggregated and analyzed by the divisional accounting personnel and then submitted to the group headquarters, which may lead to the redundancy of personnel and departments, resulting in the untimely collection of financial information from the group headquarters, operational errors and problems such as information asymmetry between online and offline. Second, there is no good communication mechanism between business information and financial information, and the core data cannot be unified and centralized in the same system for business analysis and management. The dual-track system of business and finance makes it impossible to allocate and apply enterprise resources efficiently. In addition, the value application and decision analysis of financial management cannot provide support for business development quickly and timely, and the efficiency of business execution is low.

### 4.2. Implementation of a Company's Financial Integration in the Internet Era

#### 4.2.1. Background and Significance of Implementation

With the continuous development of computer technology, approaching the “Internet” and reshaping the accounting process to break the “information silo” are undoubtedly crucial to realize the integration of business and finance of enterprises. In the background of the group's increasing business and continuous expansion, reshaping the correlation between business and finance, through the integration of business and finance, is conducive to breaking the awkward situation of information isolation of various departments, so that finance can provide timely and true feedback on business facts, and provide efficient support to the group's internal decision-making and control, to achieve “business pulling finance, finance supporting business.” The key to the integration of business and finance lies in achieving the “two-wheel drive” of finance and business. The key to the integration of business and finance lies in how to reorganize the accounting process from the group business process reorganization. The following is an example of a company's implementation path, explaining how it uses the financial sharing platform to integrate business and finance and empower management.

#### 4.2.2. Implementation Path

To realize the integration of business and finance for management empowerment, a company makes full use of the financial sharing platform. A company's financial sharing center is an integrated and unified accounting platform based on front-end business pull-through. All transactions, invoices, reconciliations, payments, and other processes in the front-end are collected as data collection points, and a large amount of data resources are collected and entered into the data platform in real-time to store the information, and the stored data are extracted, summarized, apportioned, offset and consolidated, and converted into caliber. The stored data are extracted, aggregated, apportioned, offset and consolidated, transformed, and then aggregated and displayed through the management dimension (see Figure 12).

We further analyzed the changes in different links of financial accounting operations in Figure 13.

Based on the report format and unified index system, the group establishes corresponding analysis models; creates a unified financial data and report platform; prepares financial statements; provides the group with standardized financial accounting, multi-dimensional cost and profitability analysis, and other services; and provides support for relevant information disclosure, group management, and decision-making (see Figure 14).

Based on the group's financial sharing unified data platform, the shared finance center has also built a multi-dimensional indicator analysis system, establishing multi-dimensional accountability indicators and analysis systems corresponding to main business income; profit before tax; operating net cash flow; major quality issues at the operation level, management level, and decision-making level, respectively; and using the group's big data platform for analysis and display. In Figure 15, we analyze the relationship between financial management and business management.

Based on the group's financial sharing unified data platform, the shared finance center has also built a multi-dimensional indicator analysis system, establishing multi-dimensional accountability indicators and analysis systems corresponding to main business income; profit before tax; operating net cash flow; major quality issues at the operation level, management level, and decision-making level, respectively; and using the group's big data platform for analysis and display.

After reshaping the financial process, a company's internal financial sharing center platform unified the entire process and buried information on key links, so that financial rules fully penetrate the whole process of related transactions, laying a solid data foundation for the group's later monthly reconciliation and data management analysis and improving the efficiency and timeliness of data provision. It also solves the problems of high labor cost and low enterprise value creation under the decentralized financial management model. The sharing center can also generate two sets of financial reports based on the corporate structure and management reports based on the management structure. After the integration of industry and finance, the operating budget execution report can be issued in real-time, allowing the group to monitor the specific implementation of the budget in real-time and providing strong support for group managers and decision-makers.

## 5. Conclusion

In conclusion, for enterprises, financial accounting management is crucial, and it is the basis of enterprise development, especially in the Internet era; enterprises need to strengthen the innovation of the financial accounting management mode to help meet the development needs of the times. But at present, it is difficult to adapt some enterprises' financial accounting management work to the development of the network era, and the management concept has not been updated in time. Enterprises must pay more attention to this, take reasonable decisions to optimize it, and further expand the field of financial accounting management by strengthening the construction of information technology and clarifying the outstanding problems, so that enterprises can obtain new development and improve the level of financial accounting management comprehensively.

## Figures and Tables

**Figure 1:** New model of financial accounting.

**Figure 2:** Traditional financial accounting.

**Figure 3:** Mechanism of accounting information system.

**Figure 4:** Evolution of traditional AIS.

**Figure 5:** Traditional AIS function diagram.

**Figure 6:** Functional diagram of AIS for business finance integration.

**Figure 7:** Design diagram of input and data structure flexibility.

**Figure 8:** Data flow flexible design diagram.

**Figure 9:** Business process flexibility design diagram.

**Figure 10:** Design of custom reports.

**Figure 11:** Different employees' opinions on the management upgrading of the financial accounting system.

**Figure 12:** Variable conversion model of a company under the integration of industry and finance.

**Figure 13:** The distribution of different accounting operations.

**Figure 14:** The process of preparing a unified data report of a company.

**Figure 15:** The value of financial management with business management.

**Table 1:** Table of contents.

Field name	Meaning
id	Table number
T_name	Table name
T_type	Type
Creator	Creator

## Data Availability

The experimental data used to support the findings of this study are available from the author upon request.
